# Artificial Intelligence Technology Combined with Ultrasound-Guided Needle Knife Interventional Treatment of PF: Improvement of Pain, Fascia Thickness, and Ankle-Foot Function in Patients

**DOI:** 10.1155/2022/3021320

**Published:** 2022-05-17

**Authors:** Silai Zhu, Yuli Niu, Jing Wang, Dan Xu, Yong Li

**Affiliations:** Department of Ultrasound Imaging, Wuhan Ninth Hospital, China

## Abstract

**Objective:**

To explore the effect of artificial intelligence (AI) technology combined with ultrasound-guided needle knife intervention in the treatment of plantar fasciitis (PF) on pain, fascia thickness, and ankle and foot function.

**Methods:**

A total of 130 patients with PF treated in our hospital from January 2019 to April 2021 were enrolled. The patients were randomly assigned into the control group and the study group. The control group received ultrasound-guided needle knife interventional therapy, and the study group received AI technology combined with ultrasound-guided needle knife interventional therapy. The curative effect, VAS score, plantar fascia thickness, plantar fascia elasticity score, plantar fascia blood flow index, and AOFAS score were investigated.

**Results:**

The total effective rate of the study group was higher compared to that of the control (*P* < 0.05). There exhibited no significant difference in VAS score before treatment, but the VAS score of the study group was lower compared to that of the control group at 2, 4, and 8 weeks after treatment. There exhibited no significant difference in plantar fascia thickness before treatment (*P* > 0.05), but after treatment, the plantar fascia thickness in the study group was lower compared to that in the control (*P* < 0.05). The plantar fascia thickness in the study group was lower compared to that in the control at 2, 4, and 8 weeks after treatment (*P* < 0.05). In terms of the plantar fascia elasticity score, there exhibited no significant difference before treatment (*P* > 0.05), but the plantar fascia elasticity score of the study group was lower compared to that of the control at 2, 4, and 8 weeks after treatment (*P* < 0.05). There exhibited no significant difference in plantar fascia blood flow index before treatment (*P* > 0.05), but after treatment, the plantar fascia blood flow index in the study group was higher compared to that in the control (*P* < 0.05). The plantar fascia blood flow index in the study group was higher compared to that in the control at 2, 4, and 8 weeks after treatment (*P* < 0.05). There exhibited no significant difference in the AOFAS score before treatment, but after treatment, the AOFAS score of the study group was higher compared to that of the control at 2, 4, and 8 weeks after treatment.

**Conclusion:**

Patients with PF receive AI technology combined with ultrasound-guided needle knife interventional therapy, which can effectively relieve pain and improve fascia thickness and ankle-foot function. Thus, AI technology combined with ultrasound-guided needle knife interventional therapy has the advantages of convenient operation, safety, and effectiveness, which is worthy of clinical application.

## 1. Introduction

Plantar fasciitis (PF) is defined as a common clinical acute and chronic soft tissue disease [1]. People with large amount of exercise and congenital abnormal plantar structure are the most common causes of plantar pain. Plantar fascia is an important structure to maintain the arch of foot [1]. If tension and traction are repeated for a long time, aseptic inflammation is easy to occur, and its pathological changes are plantar fascia degeneration, hypertrophy, calcification, adhesion, and contracture [2]. The periosteum at the medial process of calcaneal tubercle was overstretched, which led to the proliferation and active proliferation of chondrocytes, continuous calcification and ossification in the attachment, and bone spur was formed over a long time, resulting in chronic plantar pain [2]. Magnetic resonance imaging (MRI) and musculoskeletal ultrasonography showed abnormal thickening of the plantar fascia, local swelling and exudation in patients with PF, and osteophyte hyperplasia in the heel in a few patients [3]. In China, as a developing agricultural and manufacturing country, the incidence of PF is increasing. Because of its pain and limited activities, it seriously affects the work and life of patients and brings a certain economic burden to patients, families, and society. In the past, patients with PF were mainly given nonoperative conservative treatment, including exercise therapy, orthopedic insole decompression, or extracorporeal shock wave analgesia; however, these treatments cannot be treated fundamentally, and they have the disadvantages of more times of treatment, easy recurrence, and unsatisfactory treatment effect [4].

In recent years, small needle knife therapy has been widely employed in the treatment of PF, especially for the treatment of intractable PF [5]. The small needle knife can dredge and peel off the metatarsal fascia with hypertrophy, adhesion, and contracture, relieve the tension and contracture of the metatarsal fascia and long metatarsal ligament, release adhesion, mash and aspirate the calcified focus in the metatarsal fascia, and grind the hyperplastic bone to its passivation, which has the advantages of simplicity, convenience, cheapness, and efficiency [6]. However, the traditional needle knife does not have the visual guidance of ultrasonic images and only determines the needle angle, depth and peeling degree, and the operator's experience [7]. There are some shortcomings, such as inaccurate location of the treatment target, too much peeling, or insufficient loosening, which is very easy to cause unnecessary damage to the surrounding tissue [8]. With the development of ultrasound medicine, musculoskeletal ultrasound can accurately provide the location and qualitative judgment of soft tissue lesions and can clearly show plantar metatarsal fascia, calcaneal tubercle, long metatarsal ligament, flexor digitorum brevis, tibial nerve, posterior tibial artery, and hyperplastic bone spur [9]. PF can be diagnosed when calcaneal tubercle bone shows olecranon-like high echo, metatarsal fascia thickness exceeding 4 mm, localized thickening, hypoechoic, or calcified focus formation. Ultrasound guidance can provide a clear location and nature of the lesions, dynamically monitor the relationship between the tip of the needle and the tissue at the operation site, and visually release adhesions, smash calcified foci and suck out, etc. [10]. Furthermore, visual accurate local injection of steroids has a good effect in eliminating aseptic inflammation of soft tissue and regulating autonomic nerve dysfunction because of its strong anti-inflammatory effect [10].

At present, the application of artificial intelligence (AI) technology to PF is still in the exploratory stage. Ultrasonic image preprocessing is not only one of the important directions of AI technology in the medical field but also a very important link in image intelligent recognition. Not only clinical ultrasound doctors will be affected by echo attenuation, echo loss, sound shadow, and so on in the process of ultrasound examination. Therefore, the preprocessing of ultrasonic image in the traditional machine recognition process includes denoising, image annotation, target segmentation, and data set imbalance processing. With the progress of medicine, the application of AI technology in ultrasonic diagnosis and ultrasound-guided interventional treatment of musculoskeletal diseases has gradually become an important means of diagnosis and treatment in rehabilitation medicine, sports medicine, and pain medicine. AI technology combined with ultrasound-guided interventional therapy of PF has the advantages of good curative effect, quick effect, and good functional recovery; compared with traditional needle knife therapy, it has irreplaceable advantages and is worthy of clinical application and promotion.

## 2. Participants and Methods

### 2.1. Patient Information

A total of 130 patients with PF treated in our hospital from January 2019 to April 2021 were enrolled. The patients were randomly assigned into the control group and the study group. The control group received ultrasound-guided needle knife interventional therapy, and the study group received AI technology combined with ultrasound-guided needle knife interventional therapy. In the control group, the age was 36-67 years old, with 46.56 ± 3.42 average age, including 35 males and 30 females, while in the study group, the age was 37-68 years old, with 46.55 ± 3.93 average age, including 36 males and 29 females. There was no statistical significance in the general data of the two groups. This study was permitted by the Medical Ethics Association of our hospital, and all patients signed informed consent.

Diagnostic criteria [11]: (1) patients over 35 years old may have a history of sharp calcaneal pressure, but most of them have no history of trauma; (2) walking pain on the metatarsal surface of the heel; (3) tenderness on the metatarsal surface of the heel; (4) the metatarsal skin of the calcaneus was not red and swollen, and the skin temperature was slightly higher; (5) hyperosteogeny or spur could be seen by X-ray examination; (6) ultrasonography showed the echo change of plantar fascia, and the thickness of plantar fascia was higher than that of 4 mm.

Inclusion criteria: (1) meet the diagnostic criteria; (2) those who agree to participate in the trial, sign the informed consent form, and can receive treatment.

Exclusion criteria: (1) do not meet the diagnostic criteria; (2) ankle osteoarthritis and calcaneal pain caused by rheumatoid arthritis, ankylosing spondylitis, gout, calcaneal tuberculosis, and other bone diseases; (3) patients with severe heart and lung disease, severe diabetes, foot skin infection, fever, poor blood coagulation, and inability to cooperate with treatment and follow-up.

### 2.2. Treatment Methods

The control group received ultrasound-guided needle knife interventional therapy: the patient was in supine position, a small sandbag was placed behind the ankle, the heel was facing down, and the sole of the foot was fully exposed. Philips Epiq 5 ultrasonic diagnostic instrument with probe frequency of 5~12 MHz was employed. Before treatment, the thickness of metatarsal fascia, echo and calcification in metatarsal fascia, and bone spur in calcaneal tubercle were examined by ultrasound. Determine the needle entry point (most of the needle entry points are similar to the traditional needle knife group). After the ultrasonic probe is coated with coupling agent, the aseptic probe cover is coated, and the needle is injected into the lesion of the metatarsal fascia under real-time ultrasonic monitoring. 0.5% lidocaine 1.5 ml and triamcinolone acetonide 0.5 ml mixture 2 ml is injected to infiltrate the metatarsal fascia, and the needle tip continues downward to reach the tip of the calcaneal spur. Using the no. 4 small needle knife, the angle between the needle body and the heel plane is 60°~80°. Reach the calcification focus of metatarsal fascia or hypertrophic metatarsal fascia, follow the fascia to dredge and peel off longitudinally, then needle knife to the tip of bone spur, peel off to bone spur passivation, and then needle out. After the location of the lesion and the blood flow signal of the operation site were confirmed by ultrasound, the aseptic excipients were covered and the heel was pressurized 10 min.

The study group received AI technology combined with ultrasound-guided needle knife interventional therapy: ultrasound-guided needle knife intervention therapy as the control group, AI technology: (1) randomly rotate the picture, the rotation angle is between 0 and 20 degrees; (2) the image is translated in a random horizontal direction, and the proportion of horizontal translation is between 0 and 10%; (3) the image is translated in a random vertical direction, and the proportion of vertical translation is between 0 and 10%; (4) enlarge and reduce the picture randomly, and the ratio of magnification and reduction is between 0 and 10%; (5) randomly flip the picture horizontally, and there is a 50% chance that the picture will be flipped horizontally; (6) randomly change the brightness of the picture, which ranges from 70% to 130%. Through data enhancement, the generalization ability of the model is greatly improved and the overfitting problem is reduced.

### 2.3. Observation Index

#### 2.3.1. Curative Effect Evaluation [12]

(1) Recovery: free walking, no obvious discomfort, heel pain completely disappeared, no local tenderness; (2) obvious effect: free walking, occasional discomfort, heel pain basically disappeared, no obvious local tenderness; (3) effective: walking was slightly limited, heel pain was mild, local tenderness was mild; (4) ineffective: limited walking, heel pain, local tenderness was obvious. Total effective rate = (cured + markedly effective + effective)/total number of cases × 100%.

#### 2.3.2. Visual Analogue Scale of Pain

Pain visual analogue scale (VAS): draw a 10 cm horizontal line on the paper, one end of the horizontal line is 0, indicating no pain; the other end is 10, indicating severe pain; the middle part indicates varying degrees of pain. Let the patient draw a mark on the horizontal line according to his self-feeling, indicating the degree of pain.

#### 2.3.3. Plantar Fascia Thickness

The patients lay prone on the treatment bed with their feet hanging out of the bed, keeping the rest position of the ankle joint. The ultrasonic probe was scanned parallel to the long axis of the foot to observe the boundary of the plantar fascia. The thickness of the plantar fascia was measured at a position about 0.5 cm from the junction of the plantar fascia and calcaneus (see Figure 1). The thickness of plantar fascia was recorded before treatment and 2 weeks, 4 weeks, and 8 weeks after treatment.

#### 2.3.4. Plantar Fascia Elasticity

The treatment patients lay prone on the treatment bed with their feet hanging out of the bed to maintain the resting position of the ankle joint. The ultrasonic probe was scanned parallel to the foot axis to determine the position of the plantar fascia. Using the assisted elastic imaging mode, the quality control index is 60-80, and the elastic image and grayscale ultrasonic image of plantar fascia are displayed at the same time. Refer to the RTSE method of foreign scholar Stroud et al. to evaluate the tendon [13] to analyze the elasticity of plantar fascia: 1—blue area contains most of the display of plantar fascia; 2—green area contains most of the display of plantar fascia; 3—plantar fascia display area in addition to blue or green, there is also a small range of red (see Figure 2). The plantar fascia elasticity was recorded before treatment and 2 weeks, 4 weeks, and 8 weeks after treatment.

#### 2.3.5. Plantar Fascia Blood Flow Index

The treatment patients lay prone on the treatment bed with their feet hanging out of the bed to maintain the resting position of the ankle joint. The ultrasonic probe was scanned parallel to the foot axis to determine the position of the plantar fascia. Turn on the color energy Doppler mode, set the sampling frame size to 1 cm × 1 cm, and set the color Doppler to the maximum sensitivity without generating noise signal. Select the image with the most abundant blood flow signal in the plantar fascia, measure the area of the blood flow signal, and then divide it by 1 square centimeter to get the percentage of the blood flow signal in the area (Figure 3). The plantar fascia blood flow index was recorded before treatment and 2 weeks, 4 weeks, and 8 weeks after treatment.

#### 2.3.6. AOFAS Ankle-Hindfoot Score

The full score of AOFAS ankle-hindfoot score [14] was 100, excellent: 90-100, good: 75-89, fair: 50-74, and poor: less than 50. AOFAS ankle-hindfoot score was performed before treatment and 2 weeks, 4 weeks, and 8 weeks after treatment.

### 2.4. Statistical Analysis

SPSS 17.0 statistical software package was employed for data analysis. The counting data were compared by the *χ*^2^ test, and the measurement data were expressed by mean ± standard deviation. The overall comparison of the scores of the two groups before and after treatment employed the analysis of variance of two factors repeated measurement data, the overall comparison of the scores of each time point in the two groups employed single factor analysis of variance, and the pairwise comparison of data between the two groups or within groups employed LSD *t*-test. The difference was statistically significant (*P* < 0.05).

## 3. Results

### 3.1. Comparison of Curative Effects

First of all, we compared the curative effects of the two groups. The total effective rate of the study group was higher compared to that of the control (*P* < 0.05). All the data are shown in Table 1.

### 3.2. VAS Score Comparison

Secondly, we compared the VAS scores of the two groups; there exhibited no significant difference before treatment, but after treatment, the VAS scores of the two groups decreased, and the VAS scores of the study group were lower compared to the control at 2 weeks, 4 weeks, and 8 weeks after treatment (*P* < 0.05). All the data are shown in Table 2.

### 3.3. Comparison of Plantar Fascia Thickness

Next, we compared the plantar fascia thickness. Before treatment, there exhibited no significant difference (*P* > 0.05). The plantar fascia thickness of the study group was lower compared to that of the control at 2, 4, and 8 weeks after treatment (*P* < 0.05). All the data are shown in Table 3.

### 3.4. Comparison of Plantar Fascia Elasticity Score

Next, we compared the plantar fascia elasticity score, and there had no significant difference between the two groups before treatment (*P* > 0.05). The plantar fascia elasticity score of the study group was lower compared to that of the control at 2, 4, and 8 weeks after treatment (*P* < 0.05). All the data are shown in Table 4.

### 3.5. Comparison of Plantar Fascia Blood Flow Index

Then, we compared the plantar fascia blood flow index. Before treatment, there exhibited no significant difference (*P* > 0.05). The plantar fascia blood flow index of the study group was higher compared to that of the control at 2, 4, and 8 weeks after treatment (*P* < 0.05). The results of all the data are shown in Table 5.

### 3.6. AOFAS Score Comparison

Finally, we compared the AOFAS scores of the two groups; there was no significant difference before treatment, but after treatment, the AOFAS scores of the two groups increased, and the AOFAS scores of the study group were higher compared to those of the control at 2, 4, and 8 weeks after treatment (*P* < 0.05). All the data are shown in Table 6.

## 4. Discussion

The heel bears most of the body weight during exercise, so heel pain will bring a lot of inconvenience and pain to people's life and work [1]. PF is the most common cause of heel pain, and it is reported that 11%-15% of all foot pain patients visit for this disease [15]. The plantar fascia exists in the deep surface of the subcutaneous adipose tissue of the foot and is an important structure for maintaining the arch of the foot, including three dense connective tissues, which originate from the medial tubercle of the calcaneus and extend between the toes [15]. It has a protective effect on the muscles, blood vessels, and nerves of the foot. When the metatarsophalangeal joint is flexion, the plantar fascia is pulled to increase the arch angle of the foot. Human long-term walking, standing, running, and jumping and other movements lead to strain at the starting point of plantar aponeurosis and then degeneration, resulting in tearing, degeneration, chronic fibrous tissue inflammation, edema, and thickening of plantar fascia [16]. Therefore, PF is a syndrome of coexistence and interaction of inflammation and degeneration [16]. PF is a kind of chronic aseptic inflammation, and the age of onset is mostly between 40 and 70 years old. Obesity, standing or walking with weight for a long time, abnormal structure of foot arch, bone spur of calcaneus, and limited movement of ankle joint are all risk factors of PF [17]. The main clinical symptoms are needle-like pain on the inside of the heel when getting up in the morning or walking after a long rest, but the pain is obviously relieved after walking for a period of time; after walking for a long time, the symptom is repeated and aggravated. The pathological process of plantar fascia directly affects the severity of heel pain [18, 19]. Inflammatory factors and inflammatory manifestations such as redness, swelling, and heat were not detected in most patients with PF. PF begins slowly and can have a history of months or years. As a self-limited disease, PF gradually alleviates and disappears even without treatment within 14 months [20]. However, the pain during the onset of the disease will cause serious inconvenience and disturbance in daily activities and easily lead to other foot and ankle diseases. Finally, there are still 10% of patients whose symptoms worsen because they are insensitive to these treatments and develop into plantar fascia disease with chronic hyaline degeneration, which requires surgical intervention [21].

At present, the common clinical treatments for PF mainly include painkillers, physiotherapy, orthopedic insole and nocturnal splint application, injection therapy, extracorporeal shock wave therapy, and surgical treatment [17]. Clinical trials show that these treatments can achieve certain clinical effects, but there are still some side effects, so if a more safe and effective method can be found, economical and convenient treatment is of great significance for patients with PF [18]. Traditional nonoperative conservative treatments such as exercise therapy, orthopedic insole decompression, or extracorporeal shock wave analgesia have the disadvantages of more times of treatment, easy recurrence, and unsatisfactory treatment effect [4]. At present, patients with refractory PF with poor effect of conservative treatment are often treated with small needle knife [22]. The small needle knife can dredge and peel off the hypertrophy, adhesion, and contracture of the plantar fascia, relieve the tension and contracture of the metatarsal fascia and long metatarsal ligament, release the adhesion, and mash and aspirate the calcified focus in the plantar fascia, which has the advantages of simplicity, convenience, cheapness, and efficiency [22]. Because of the uniqueness of the design of small needle knife, it has two different action mechanisms of needle and knife, which can not only activate meridians and acupoints by stimulating local meridians and acupoints but also exfoliate adhesion and release contracture of diseased soft tissue [23]. Needle knife treatment can improve the blood circulation of the injured site and promote fibrin exudation through peeling and release, which can effectively relieve pain and accelerate local tissue repair. According to the framework of “bowstring theory” and “mesh theory,” PF belongs to chronic soft tissue injury at the starting and ending point of foot soft tissue [5]. Therefore, needle knife therapy can effectively relieve the pain symptoms of patients with PF and restore the normal biomechanical balance and normal physiological function of the foot which is generally accepted by patients, and its clinical effect is also recognized by most clinicians.

The core of the pathological pathogenesis of needle knife medicine is the theory of imbalance between yin and yang, including the theoretical system of mechanical balance, anatomical balance, and metabolic balance [24]. The main purpose of needle knife therapy is to regulate, restore, or even reconstruct these balances, so as to have a therapeutic effect on diseases. Needle knife medicine regards the course of human chronic soft tissue injury as a whole and each stage of the course as a part of the whole course [24]. The overall concept of needle knife medicine is mainly as follows: (1) the human body is the structural whole of mechanics: because the human body is the life body of complex mechanical mechanism and structure, the change of the structure of the mechanical mechanism of any human body in this whole will directly affect the change of the structure of the human body, which may lead to the imbalance of the human body, and the needle knife medicine adjusts the structure of the human body. (2) The human bowstring mechanical system is an important morphological basis for studying the overall mechanical mechanism of the human body: the human bowstring system is the system connecting the mechanical relationship between human bone and soft tissue. The abnormal force of the human bowstring system is the main cause of chronic soft tissue injury. When the human body cannot compensate for this abnormal stress, it may lead to the clinical symptoms of chronic soft tissue injury. (3) The mesh theory is the overall pathological framework of human chronic soft tissue injury: the mesh theory holds that chronic soft tissue injury is not a simple local lesion, but an overall pathological framework with points and lines [24].

Furthermore, needle knife medicine makes the needle knife treatment of local lesions jump to the height of the treatment of the whole pathological framework [25]. Under the guidance of the whole scientific theory of traditional needle knife medicine, needle knife treatment pays attention to the integrity of human chronic soft tissue injury, and needle knife medical treatment is carried out under nondirect vision conditions. The adhesion and contracture of each part of the key lesion were cut and separated, and the three-dimensional and network-like pathological structure of each part of the lesion was destroyed [23]. As a result, the mechanical anatomical system and the overall mechanical equilibrium of the bow string in each part of the lesion gradually returned to normal. Thus, it can play a role in preventing and treating various diseases. Small needle knife is a kind of therapy produced on the basis of Chinese traditional nine needles, combined with acupuncture meridians and modern anatomy [25]. With the development and maturity of basic theories such as “bow string theory” and “mesh theory,” needle knife has been widely employed in clinical practice, and the curative effect has been affirmed by the majority of clinical workers and patients.

In the past, the clinical diagnosis of PF was mainly based on medical history and physical examination. In recent years, with the development of ultrasound medicine, musculoskeletal ultrasound has become the objective, rapid, and reliable first choice for early diagnosis of PF [26]. The normal plantar fascia showed a uniform echo band structure located in the calcaneal tubercle covering the surface of the plantar muscle with a thickness < 4 mm. Plantar PF can be diagnosed when ultrasound shows localized thickening with decreased echo. Ultrasonic diagnosis of PF is effective and reliable [26]. With the development of ultrasound medicine, musculoskeletal ultrasound can accurately provide the location and qualitative judgment of soft tissue lesions and can clearly show plantar metatarsal fascia, calcaneal tubercle, long metatarsal ligament, flexor digitorum brevis, tibial nerve, posterior tibial artery, and hyperplastic bone spur and its relationship with adjacent tissues. Ultrasound guidance can provide a clear location and nature of the lesions, dynamically monitor the relationship between the tip of the needle and the tissue at the operation site, and visually release adhesions, smash calcified foci and suck out, etc. it avoids the problems of inaccurate location of the target area, too much peeling or insufficient loosening in the traditional needle knife, and avoids unnecessary damage to the surrounding tissue.

However, in the process of practical application, due to the lack of quantitative measurement of image features and the difference of people's visual perception, the visual evaluation under the guidance of ultrasound is time-consuming, and the accuracy is still affected by the doctor's clinical experience [9]. With the development of AI in the medical field, more AI technologies are applied in medical intelligence decision diagnosis. Deep learning technology is the most mainstream technology in the field of AI medical imaging, in ultrasound-guided auxiliary diagnosis and interventional therapy [27]. Image preprocessing is a very important part of intelligent image recognition. Medical ultrasound images are easily affected by echo attenuation and speckle noise, which leads to poor image quality, which not only interferes with observer analysis and diagnosis but also affects the effect of feature extraction, analysis, and classification in the process of image recognition by computer [27]. In the research of ultrasonic image denoising, Johannsen et al. carry on wavelet transform to the image, denoise the second layer component of the detail through the soft closed value, and then improve the image quality through the anisotropic diffusion model [28]; Lee et al. [29] use adaptive weighted median filter (AWMF) to denoise the ultrasonic image; Asheghan et al. [30] denoise the image by improving the Savitzky-Golay filter. Abdullah et al. [31] put forward various data processing methods such as unbalanced data preprocessing, sampling method, and unbalanced data cleaning. In a word, the ultrasonic analysis technology under the blessing of AI has played a very obvious role in improving the diagnosis rate.

In conclusion, patients with PF receive AI technology combined with ultrasound-guided needle knife interventional therapy, which can effectively relieve pain and improve fascia thickness and ankle-foot function. Thus, AI technology combined with ultrasound-guided needle knife interventional therapy has the advantages of convenient operation, safety, and effectiveness, which is worthy of clinical application. However, our research also has some shortcomings, such as the number of cases is not enough and the follow-up time is not long enough. Therefore, our conclusions need to be confirmed by more case studies.

## Figures and Tables

**Figure 1:** Measurement of plantar fascia thickness at about 0.5 cm from the junction of plantar fascia and calcaneus.

**Figure 2:** Plantar fascia elasticity score: using the booster mode, the quality control index is 60-80. The left side shows the B-mode ultrasound image, and the right side shows the elastic image. (a) The blue area contains most of the display of the plantar fascia; (b) the green area contains the display of most of the plantar fascia; (c) the area of the plantar fascia is shown in addition to blue or green.

**Figure 3:** Plantar fascia blood flow index: measure the area of the blood flow signal at the plantar fascia in the figure and then divide it by 1 square centimeter to get the percentage of the blood flow signal in the area.

**Table 1:** Comparison of nursing satisfaction (*n*/%).

Group	*N*	Cure	Significant effect	Effective	Invalid	Total efficiency
C group	65	45 (69.23)	8 (12.31)	7 (10.77)	5 (7.69)	60 (92.31)
R group	65	53 (81.54)	11 (16.92)	1 (1.54)	0	65 (98.46)
*χ* ^2^						5.200
*P*						0.022

**Table 2:** Comparison of VAS scores between the two groups ($\bar{x}\pm s$, points).

Group	*N*	Before treatment	2 weeks after treatment	4 weeks after treatment	8 weeks after treatment
C group	65	7.48 ± 0.24	5.63 ± 0.53	3.86 ± 1.23	2.84 ± 0.64
R group	65	7.41 ± 0.44	4.66 ± 1.34	2.46 ± 0.31	1.22 ± 0.12
*t*		1.126	5.427	8.898	20.058
*P*		0.262	<0.001	<0.001	<0.001

**Table 3:** Comparison of plantar fascia thickness ($\bar{x}\pm s$, mm).

Group	*N*	Before treatment	2 weeks after treatment	4 weeks after treatment	8 weeks after treatment
C group	65	5.38 ± 0.56	5.04 ± 0.53	4.81 ± 0.32	4.10 ± 0.35
R group	65	5.31 ± 0.52	4.81 ± 0.42	4.03 ± 0.53	3.56 ± 0.56
*t*		0.738	2.742	10.157	6.592
*P*		0.461	<0.001	<0.001	<0.001

**Table 4:** Comparison of plantar fascia elasticity scores between the two groups ($\bar{x}\pm s$, points).

Group	*N*	Before treatment	2 weeks after treatment	4 weeks after treatment	8 weeks after treatment
C group	65	2.79 ± 0.76	2.69 ± 0.33	2.23 ± 0.36	1.38 ± 0.45
R group	65	2.71 ± 0.57	2.21 ± 0.21	1.36 ± 0.31	1.16 ± 0.21
*t*		0.678	9.893	14.764	3.571
*P*		0.498	<0.001	<0.001	<0.001

**Table 5:** Comparison of plantar fascia blood flow index between the two groups ($\bar{x}\pm s$).

Group	*N*	Before treatment	2 weeks after treatment	4 weeks after treatment	8 weeks after treatment
C group	65	3.58 ± 0.44	4.58 ± 0.63	4.59 ± 0.46	4.53 ± 0.75
R group	65	3.51 ± 0.38	5.53 ± 0.42	5.06 ± 0.52	5.05 ± 0.72
*t*		0.970	10.115	5.457	4.032
*P*		0.333	<0.001	<0.001	<0.001

**Table 6:** Comparison of AOFAS scores between the two groups ($\bar{x}\pm s$, points).

Group	N	Before treatment	2 weeks after treatment	4 weeks after treatment	8 weeks after treatment
C group	65	60.48 ± 5.23	66.79 ± 3.42	74.67 ± 4.42	83.93 ± 3.33
R group	65	60.49 ± 5.22	70.48 ± 3.31	80.83 ± 4.21	87.83 ± 4.31
*t*		0.010	6.250	8.136	5.772
*P*		0.991	<0.001	<0.001	<0.001

## Data Availability

No data were used to support this study.

## References

[1] Qin Z., Bo Y., Xinghua L. (2021). Clinical observation of exercise bandage technique combined with extracorporeal shock wave in the treatment of PF. *Chinese Journal of Rehabilitation Medicine*.

[2] Patrick W. C., Chloe D. (2021). Similar benefits seen after radial extracorporeal shockwave therapy or autologous blood injection in patients with chronic PF—a retrospective cohort study. *Clinical Journal of Sport Medicine*.

[3] Fei X., Lang L., Lingjiao H., Wei C., Zhou X. (2021). Platelet-rich plasma has better mid-term clinical results than traditional steroid injection for PF: a systematic review and meta-analysis. *Orthopaedics & Traumatology: Surgery & Research*.

[4] Sulithep P., Rotsalai K., Praneet P. (2021). Immediate and short-term effects of kinesiotaping and lower extremity stretching on pain and disability in individuals with PF: a pilot randomized, controlled trial. *Physiotherapy Theory and Practice*.

[5] Baur D., Schwabl C., Kremser C. (2021). Shear wave elastography of the plantar fascia: comparison between patients with PF and healthy control subjects. *Journal of Clinical Medicine*.

[6] Melese H., Alamer A., Getie K., Nigussie F., Ayhualem S. (2021). Extracorporeal shock wave therapy on pain and foot functions in subjects with chronic PF: systematic review of randomized controlled trials. *Disability and Rehabilitation*.

[7] Pavinee H., Sujitra B., Praneet P. (2021). Differences in lower-extremity kinematics between the male military personnel with and without PF. *Physical Therapy in Sport*.

[8] Jiang Hai Y. Y., Zhicheng L., Qiliang Z. (2021). Extracorporeal shock wave and corticosteroid injection in the treatment of PF: comparison of plantar pressure and gait analysis. *Research on tissue Engineering in China*.

[9] Ozdemir Y. B., Atan T. (2021). Effects of adjuvant low-dye Kinesio taping, adjuvant sham taping, or extracorporeal shockwave therapy alone in plantar fasciitis: a randomised double-blind controlled trial. *International Journal of Clinical Practice*.

[10] Dinkar K. S., Kapoor R., Mishra V. K., Pal C. P., Sharma M., Yadav R. (2021). Role of platelet-rich plasma in painful early osteoarthritis knee and PF: a prospective study. *Journal of Orthopedics, Traumatology and Rehabilitation*.

[11] Goel N., Talwar J., Agarwal S., Krishna L. G., Rustagi A. (2021). A comparative study between intralesional platelet rich plasma injection and extracorporeal shockwave therapy for the treatment of PF. *Journal of Arthroscopy and Joint Surgery*.

[12] Lee J. H., Jung H. W., Jang W. Y. (2020). A prospective study of the muscle strength and reaction time of the quadriceps, hamstring, and gastrocnemius muscles in patients with PF. *BMC Musculoskeletal Disorders*.

[13] Stroud W., Alexander B., Halstrom J. R. (2020). Outcomes of gastrocnemius recession in patients with PF and Achilles tendinosis:a retrospective study of 160 patients. *Foot & Ankle Orthopaedics*.

[14] Yicen Z., Peixin W., Zhicheng L. (2021). Ultrasound-guided injection of sodium hyaluronate and corticosteroids in the treatment of PF: pain, fascia thickness and ankle-foot function evaluation. *Research on tissue Engineering in China*.

[15] (2020). Efficacy of acupuncture versus sham acupuncture or waitlist control for patients with chronic plantar fasciitis: study protocol for a two-centre randomised controlled trial. *BMJ Open*.

[16] Mills K. M., Preston E. B., Choffin Schmitt B. M. (2020). Embedding pain neuroscience education in the physical therapy management of patients with chronic PF: a prospective case series. *Journal Of Manual & Manipulative Therapy*.

[17] Erden T., Toker B., Cengiz O., Ince B., Asci S., Toprak A. (2020). Outcome of corticosteroid injections, extracorporeal shock wave therapy, and radiofrequency thermal lesioning for chronic PF. *Foot & Ankle International*.

[18] Armagan Alpturker K., Cerrahoglu A. B. L., Orguc I. S. (2020). Evaluation effects of laser therapy and extracorporeal shock wave therapy with clinical parameters and magnetic resonance imaging for treatment of PF in patients with spondyloarthritis: a randomized controlled trial. *International Journal of Rheumatology*.

[19] Purnima A., Vivek J., Garg S. K. (2020). Evaluation of plantar fascia using high-resolution ultrasonography in clinically diagnosed cases of PF. *Polish Journal of Radiology*.

[20] Bagcier F., Yilmaz N. (2020). The impact of extracorporeal shock wave therapy and dry needling combination on pain and functionality in the patients diagnosed with plantar fasciitis. *The Journal of Foot and Ankle Surgery*.

[21] Heide M., Mørk M., Røe C., Brox J. I., Hoksrud A. F. (2020). The effectiveness of radial extracorporeal shock wave therapy (rESWT), sham-rESWT, standardised exercise programme or usual care for patients with plantar fasciopathy: study protocolfor a double-blind, randomised, sham-controlled trial. *Trials*.

[22] Lei X., Yanning K., Xinglu H., Pingbo L., Dingzhang C., Jichao Y. (2019). Preliminary study on quantitative evaluation of traditional Chinese medicine bone-rectifying manipulation in the treatment of chronic PF by ultrasonic elastography. *Journal of Clinical Ultrasonic Medicine*.

[23] Ping L., Donghai W., Fangfang G., Dani W. (2019). Clinical value of ultrasound-guided treatment of PF. *Chinese Journal of Medical Imaging*.

[24] Hao C., Weiping L., Xianzhong G., Chenjie X., Hua G., Hongguang B. (2018). Observation on the efficacy of ultrasound-guided platelet-rich plasma injection in the treatment of PF. *Journal of Clinical Anesthesiology*.

[25] Ping L., Xingguo W., Donghai W., Fangfang G., Dani W. (2018). Anatomical characteristics of plantar aponeurosis were analyzed by ultrasonic shear wave elastography and multimodal imaging. *Research on tissue Engineering in China*.

[26] Xiulin H., Ketao W., Xiaoying Z. (2018). Prognostic analysis of PF treated with barometric ballistic shock wave and ultrasound-guided steroid interventional therapy. *Journal of Southern Medical University*.

[27] Huang K., Giddins G., Wu L. D. (2020). Platelet-rich plasma versus corticosteroid injections in the management of elbow epicondylitis and plantar fasciitis: an updated systematic review and meta-analysis. *The American Journal of Sports Medicine*.

[28] Johannsen F., Konradsen L., Herzog R., Krogsgaard M. R. (2020). Endoscopic fasciotomy for PF provides superior results when compared to a controlled non-operative treatment protocol: a randomized controlled trial. *Knee surgery, sports traumatology, arthroscopy : official journal of the ESSKA*.

[29] Lee D. O., Yoo J. H., Cho H. I., Cho S., Cho H. R. (2020). Comparing effectiveness of polydeoxyribonucleotide injection and corticosteroid injection in PF treatment: a prospective randomized clinical study. *Foot and Ankle Surgery*.

[30] Asheghan M., Hashemi S. E., Hollisaz M. T., Roumizade P., Hosseini S. M., Ghanjal A. (2020). Dextrose prolotherapy versus radial extracorporeal shock wave therapy in the treatment of chronic PF: a randomized, controlled clinical trial. *Foot and Ankle Surgery*.

[31] Alotaibi A., Petrofsky J., Daher N. S. (2020). The effect of monophasic pulsed current with stretching exercise on the heel pain and plantar fascia thickness in plantar fasciitis: a randomized controlled trial. *Healthcare*.

